The article "An Atypical Pleomorphic Lipomatous Tumor Presenting As Groin Mass" was published in 2021. Journal: Cureus.

# An Atypical Pleomorphic Lipomatous Tumor Presenting As Groin Mass

**DOI:** 10.7759/cureus.19410

**Published:** 2021-11-09

**Authors:** Egon Rodrigues, Florinda Cardoso, Horácio Scigliano, Mário Nora

**Affiliations:** 1 General Surgery, Centro Hospitalar de Entre Douro e Vouga, Santa Maria da Feira, PRT; 2 Anatomical Pathology Laboratory Dr. Albino Oliveira (Unilabs), Centro Hospitalar de Entre Douro e Vouga, Santa Maria da Feira, PRT

**Keywords:** soft-tissue tumor, groin mass, adipocytic tumor, atypical spindle cell/pleomorphic lipomatous tumor, atypical pleomorphic lipomatous tumor

## Abstract

Cutaneous tumors with adipocyte differentiation are frequently excised by surgeons in their daily clinical practice and sometimes less common histological diagnoses arise. Knowledge of different pathological entities and their natural history is essential for better patient management.

Atypical spindle cell/Pleomorphic lipomatous tumor (ASPLT) is a recent group included in the WHO classification. We report a case of a middle-aged man with an atypical pleomorphic lipomatous tumor in an unusual location.

## Introduction

Adipocytic tumors are the most common soft-tissue tumors, and surgical removal of these lesions is a procedure widely performed in general surgery. In 2020, WHO published a new classification of Soft Tissue and Bone Tumours, differentiating several entities [1]. The atypical spindle cell/pleomorphic lipomatous tumor (ASPLT) was included as an entity for the first time in this edition. Although it is considered a rare subtype [2,3], its incidence has not yet been described.

We report the case of an atypical pleomorphic lipomatous tumor that presented as a rapidly enlarging mass in the right groin region.

## Case presentation

A 58-year-old man, with no relevant medical history, presented with a history of an enlarging painless mass at his right groin region for the past three months (Figure 1). The patient did not have any other complaints or symptoms. Physical examination revealed a firm, skin-colored and mobile tumor with well-defined margins (5 cm largest diameter). There were no palpable adenomegalies.

**Figure 1:** Mass in the right groin region.

The patient was referred to the General Surgery department by a urologist, with suspicion of a soft-tissue tumor. An MRI described a “focal subcutaneous lesion with nodular morphology of 4.7 cm and no malignancy features”. Based on clinical and image findings, it was decided to perform an excisional biopsy.

Despite the apparent benign characteristics, the lesion was surgically removed along with the surrounding adipose tissue, preserving the margins. There were no complications related to the procedure.

Grossly, it was a subcutaneous nodular non-capsulated solid lesion, multilobulated, well-circumscribed, greyish-yellowish, without necrotic areas (Figure 2). Microscopically, a variable amount of atypical bland spindle cells and mature adipocytes were seen, with multinucleated floret-like cells in a myxoid stroma with ropey collagen bundle cells. Sclerosing areas were not disclosed (Figure 3). On immunohistochemistry, the tumor was stained for CD34, S100, and MDM2 (focal-weak), whereas CDK4 expression was absent (Figure 4). Based on these findings, an atypical pleomorphic lipomatous tumor was diagnosed.

**Figure 2:** Gross aspect of the tumor.

**Figure 3:** H&E stain.

**Figure 4:** Immunocytochemistry of (A) CD34; (B) S100; and (C) MDM2.

## Discussion

Cutaneous tumors with adipocyte differentiation are frequently excised by surgeons. Although they are mostly lipomas or angiolipomas, other rare entities can arise and raise doubts. Recently, WHO published the 5^th^ edition of soft-tissue tumors classification which included a new group, the atypical spindle cell/pleomorphic lipomatous tumor (ASPLT) [1].

Mentzel T et al. proposed the term “atypical spindle cell lipoma” for the first time in 2010 [4], suggesting that these neoplasms most likely represent an independent entity closely related to spindle cell lipoma rather than a morphologic variant of atypical lipomatous tumor/well-differentiated liposarcoma [4]. Since then, other works have given strength to this theory [2,5-7], representing now a newly established diagnostic entity [1].

ASPLT is a morphologic spectrum of benign adipocytic neoplasms [1]. The cellularity of the tumors is the basis of the spectrum. At one end, tumors can be paucicellular with few atypical spindle cells and abundant extracellular matrix. At the other extreme, they may be significantly more cellular, with less extracellular matrix [8]. As result, there is a wide range of microscopic appearance of ASPLT due to the extremely variable proportions of spindle cells, adipocytes, lipoblasts, and extracellular matrix [1]. Our case represents an atypical pleomorphic lipomatous tumor characterized by the presence of floret-like multinucleated giant cells [7].

This entity can affect both sexes, with a slight male predominance, including mostly middle-aged adults with a peak in the sixth decade [1], likewise our patient. Unlike classic spindle cell/pleomorphic lipomas, ASPLT has a wide anatomical distribution [7] and the clinical differential diagnosis depends on the involved location. The most common locations are the extremities [1]. Abdominal wall and groin areas are infrequent locations. Literature search [2-7, 9-16] shows that Bahadır B et al. [2] and Anderson WJ et al. [9] each described a case in the groin region. Also, two more cases were described on the abdominal wall [2] and Mariño-Enriquez A et al. [6] described 15 cases on the trunk, not specifying the affected regions.

For palpable lesions, ultrasound can be used in the initial investigation, but MRI remains the imaging gold standard [17]. Our patient already had an MRI report, so further diagnostic imaging evaluation was not necessary. Although the MRI favored the presence of a benign soft-tissue tumor, the rapid growth and size raised concerns about its etiology. Johnson CJ et al. found that tumor depth, a size larger than 5 cm, and history of rapid growth were the most sensitive markers of malignancy [18]. When technically possible and available, a core needle biopsy can be performed for histological examination, particularly if a sarcoma is the main suspicion [19]. However, it is not mandatory, especially when tumors are superficial. In this case, we chose to perform an excisional biopsy given the easy access and since our main suspicion was a benign tumor. Nevertheless, the lesion was removed with gross margins preserved, as it did not cause greater aesthetic or functional damage. Frozen section diagnosis and fine-needle aspiration are generally not recommended.

Histological differential diagnosis of ASPLT is highly dependent on the predominant histological features of each tumor. This entity can be considered a category between classic spindle cell/pleomorphic lipoma and liposarcoma, namely: WDL (also designated atypical lipomatous tumors) or pleomorphic liposarcoma (PLS) in cases with significant pleomorphism [2]. In dubious situations, immunohistochemistry and/or molecular tests can be carried out. In ASPLT, the neoplastic cells frequently express CD34, S100, and desmin, whereas MDM2 and CDK4 expression are rare. Expression of MDM2 or CDK4 can be seen in 5% of cases, but always in the absence of corresponding gene amplification. Simultaneous MDM2 and CDK4 expression has never been described [8]. In the present case, the tumor was stained for CD34 and S100 (desmin was not evaluated). There was also a focal and weak expression of MDM2, while CDK4 expression is absent.

Regarding the differential diagnosis of malignancy, PLS can involve the dermis or subcutaneous tissue in 25% of cases. Most patients report a rapidly growing painless mass (median: 3-6 months) [1], similar to our case. However, it is characterized by a large size, greater pleomorphism, high mitotic activity, and tumor necrosis. Our findings, such as floret-like multinucleated cells, are typical of ASPLT instead of PLS [6]. WDL is a locally aggressive tumor with a risk of dedifferentiation, which appears most often in the proximal extremities and the retroperitoneum [1]. Terminology of atypical lipomatous tumor or WDL primary depends on tumor’s location and relates to its resectability [8]. These tumors affect adults within the same age range as ASPLT. They may be morphologically indistinguishable from fat-rich ASPLT but can be distinguished by MDM2/CDK4 immunohistochemistry or by molecular testing for MDM2 gene amplification [8].

Regarding benign differential diagnosis, classic spindle cell/pleomorphic lipoma are capsulated lesions with no atypia [6], that are immunohistochemical similar to ASPLT. The distinction between this entity and an ASPLT with focal atypia can be extremely difficult. If the lesion appears on the posterior neck and shoulder, then classic spindle cell/pleomorphic lipoma is most likely [8]. Unlike ASPLT, the recurrence rate is low [1]. Other differential diagnoses are angiofibroma and myofibroblastoma, nodular CD34+ neoplasms like ASPLT, which have an anatomical preference for the groin area. In general, these two entities show a less-prominent fat component, mainly consisting of spindle cells with a hyalinized stromal background [20].

Complete surgical excision (i.e., lesion-free margin) is the appropriate treatment for ASPLT. Incompletely removed lesions may locally recur in 10-15% of the cases [1]. In cases of incomplete excision, widening of the margins or patient follow-up for a possible local recurrence seem suitable options. There is no need for regular imaging control. To the best of our knowledge, there is no risk for metastasis [1], hence there is no role for adjuvant treatment.

## Conclusions

When a soft-tissue tumor is suspected, a diagnostic approach may include an ultrasound or an MRI and eventually a core needle biopsy. The diagnosis of ASPLT can be challenging and the morphological differential diagnostic range can be broad due to the wide variety of microscopic appearances. Recognition of morphologic clues and immunohistochemistry/molecular tests to confirm the diagnosis and exclude WDL and PLS are crucial. Although it is a benign adipocytic tumor, it carries a considerable risk of local recurrence.
